RETRACTED

# Model Construction of College Students' Entrepreneurial Ability Cultivation in Mental Health Education Environment

**DOI:** 10.1155/2022/7550792

**Published:** 2022-08-19

**Authors:** Muqian Huang

**Affiliations:** School of Education, South China Normal University, Guangzhou 510000, China

## Abstract

National policies have been very supportive of college students as a new force in IEE (innovation and entrepreneurship education). Universities across the nation have increased their emphasis on entrepreneurship education and put a lot of effort into developing and enhancing college students' EA (entrepreneurship ability). An important challenge facing universities is how to develop the psychological quality of IEE in college students and create a long-term training system. The author develops the EA evaluation model for college students based on practical experience with mental health education and applies BPNN (BP neural network) theory to the assessment of IEE in higher education. The scores corresponding to the students' evaluation indices are used as input vectors, and the innovative EA of the students is evaluated. According to the simulation's outcomes, the number of hidden neurons is calculated, and the outcomes are assessed through experiments. The outcomes demonstrate that, following the completion of the enhanced BPNN training, the actual value is valid, the expected value is reasonable, and the maximum relative error between them is 1.6 percent, which is essentially the ideal situation. It has been established that the IEE's established evaluation index system is fair and can accurately capture students' IEE spirit.

## 1. Introduction

Business practice demonstrates that innovation is the unending source of national development and the constant force behind modern development [1]. Practice demonstrates that IEE (innovation and entrepreneurship education) activities are more of a psychological aptitude test for students, and psychological aptitude is a crucial component of IEE activities' success. The psychological quality of IEE education for college students could be considered the centre of university IEE. The study of educational and teaching subjects' psychological behaviours as well as the processes and rules governing their growth and change is known as educational psychology. The complete integration of educational psychology theory into college students' IEE and creation of a new educational model are of major theoretical and practical significance for the development of IEE.

As the subject of IEE, college students' reaction and psychological changes are closely related to the external environment, especially university education. On the one hand, college students' self-employment can solve the problem of the shortage of jobs provided by the society; on the other hand, it can contribute to China's economic and industrial transformation. At present, domestic scholars have a relatively consistent understanding of the problems existing in the development of business education in university in China, first of all, the problems existing in university. For example, Su and others thought that the idea of university education is backward, which limits the development of students, mainly reflected in the cognitive bias of university administrators [2]. Grichnik et al. thought that universities should set up entrepreneurial research institutions, promote the project operation of entrepreneurship, actively organize students to participate in employment and entrepreneurship knowledge competitions, entrepreneurial plan competitions, and entrepreneurial surveys of college students, vigorously support the construction of entrepreneurial associations, and comprehensively carry out entrepreneurial practice activities [3]. Bond et al. discussed the relationship between entrepreneurship education and quality education, put forward an educational model suitable for Chinese universities, analyzed the necessary elements of this new model of entrepreneurship education, and finally put forward the development countermeasures of entrepreneurship education in Chinese universities [4]. As entrepreneurship education started late in China, so far, the theory of entrepreneurship education in China is still in the discussion stage, lacking empirical analysis, and the theoretical system has not yet formed.

RETRACTED

Whether it is IEE or mental health education, its implementation, impact, and improvement are closely related to teachers' teaching levels. It is imperative that students receive psychological education in order to develop their personalities and to help them develop entrepreneurial values and qualities. It includes not only the innate foundation but also the learned environmental influence, the outcome of study, and training. The school and the government can take action for college students' business education and lay a solid foundation for the reform and innovation of education and teaching through research into college students' business education, exploring the issues at hand and looking for solutions. They can create a platform for the campus environment that encourages innovation and aids in practice training so that traditional scientific research, teaching responsibilities, and university economic development can all be better integrated. It is helpful for quickly raising college students' entrepreneurial ability and more effectively putting China's innovation-driven development strategy into practice [5].

RETRACTED

### 1.1. Research Innovation

1. This study combines quantitative research with qualitative research and uses relevant data at the microlevel to build an EA evaluation model for college students, which can provide some reference for other universities to conduct EA evaluation for college students.
2. BPNN model is a new idea to study IEE, which can improve the quality of students' IEE by establishing a scientific evaluation index system. The collected data are used to train BPNN, and the weights and thresholds of the neural network are constantly adjusted until the standard error requirements are met, and the real output value is compared with the expected output value.

## 2. Related Work

### 2.1. Research on EA of College Students

EA differs from general ability in that it is a comprehensive skill related to social occupation and that it also carries a wealth of connotations. This book asserts, based on the existing literature, that EA of college students refers to those who have recently graduated from college but have not found employment through the education of school, society, family, and other sources, with the capacity to effectively translate corporate vision into reality and to integrate resources to generate greater value.

Kwg et al. thought that EA is a psychological activity function with strong comprehensiveness and creativity, which is centered on people's intellectual activities. It is a psychological process that is closely combined with individual psychological tendencies and characteristics, formed and played a role under the restriction and influence of personality [6]. Liu et al. thought that EA is a practical ability, a kind of ability with strong comprehensive degree, a kind of creative ability, and a kind of creativity with self-development and self-realization [7]. It is considered that EA is the main psychological condition to promote the successful development of entrepreneurial activities. This psychological function has strong comprehensiveness and creativity and some congenital factors, but it is also a behavior formed by the accumulation of individual knowledge, experience, and skills, which can be manifested in entrepreneurial practice [8].

Dong et al. believed that college students' EA elements include professional skills, market control, business management, and some comprehensive abilities [9]. Lucas and others thought that the element system of EA is mainly composed of four levels: consciousness, knowledge and skills, organization and management, and opportunity discrimination and insight [10]. Yao et al. put forward a training model aimed at promoting innovation and EA [11]. Zhu selected students with entrepreneurial enthusiasm, guided them to form their own creative plans, simulated entrepreneurial implementation through feasibility, business plans, and emergency paths, and finally evaluated the results [12].

RETRACTED

### 2.2. Research Status of College Students' EA Evaluation

There are four main directions in the domestic academic research on college students' EA, namely, the connotation and measurement of EA, influencing factors, training path and promotion strategy, and evaluation system. Lin et al. analyzed the connotation and elements of EA and established a three-tier index system. The first-level index consists of four dimensions: innovation, opportunity, leadership, and risk tolerance [13]. Zhang et al. put forward multidimensional extension matter-element model and extension evaluation method to evaluate college students' EA based on extension matter-element theory and extension set theory [14]. Cai and Kong put forward that the goal of IEE is vocational ability and learning ability, and completing students' ambition is the ultimate goal of IEE [15]. Jiang and Wang integrated IEE courses into multidisciplines, wide fields, and various levels, covering management, social capital, law, financial accounting, marketing, team building, and personal quality and ability [16].

Zhang et al. thought that the responsibility of university in the new era is to enhance students' entrepreneurial awareness and EA and guide students to learn the skills of market operation in a reasonable curriculum system under the guidance of correct objectives, so as to enhance their ability to start their own businesses [17]. He et al. believed that the emergence of innovative education is an educational idea accompanied by the rise of knowledge economy. This educational idea is based on creation, aiming at cultivating innovative spirit in students' consciousness, ability, and personality [18]. Tseng and Luo set out from the connotation direction of ability and constructed an evaluation index system including three first-level indexes: scientific research quality, participation ability, and research results [19]. Guo et al., according to the problems existing in the traditional evaluation methods, used naive Bayesian network clustering method to evaluate the ability. On the basis of useless label classification, they can also refine rules and predict the ability value, effectively improving the accuracy of prediction [20].

## 3. Methodology

### 3.1. Establishment of EA Quality Model for College Students

IEE awareness is a person's interest in and need for IEE practices. It is the “initiator” and “engine” of entrepreneurship activities, encouraging and motivating people to engage in IEE practice. College mental health and IEE courses do not mesh well together. It follows that including mental health education in the IEE curriculum will help students' psychological well-being. College students score highly in the business knowledge and interpersonal skills domains of the innovation EA, but they struggle in the leadership, adaptability, and leadership domains. In terms of entrepreneurship policy funding, we should appropriately increase the financial support for college students' entrepreneurial projects through the design of an innovation fund that complies with the demands of entrepreneurship education; enable teachers to industrialise scientific and technological advances through external transfer, cooperative transformation, capital investment, and self-employment; improve the distribution mechanisms for scientific and technological advancements and income distribution.

RETRACTED

There are two levels of influence that are constant and have a significant impact: the level of personal quality and the level of the social context. In other words, whether we cultivate EA for college students or not, individual quality and social environment exist objectively or promote or hinder the formation and development of EA. China's IEE infrastructure has generally been behind, and it needs to be strengthened. We should think about how to create fundamental platforms in the future, like big data and innovative, entrepreneurial infrastructure, so that these auxiliary forces can actually provide the fundamental support they promise. The output of the upper neuron is used as the input of the lower neuron in an artificial neural network, and information is transmitted back and forth between the two neurons. Deep learning can create a depth model with multiple hidden layers, enhance the model's generalisation, and automatically learn more useful features from vast amounts of unsupervised training data, according to the state of the research on the technology. Since only word vectors are used as input features, the deep learning method is used in this paper to build the deep evaluation object extraction model.

The hidden layer of the stacked automatic encoder model is constructed by unsupervised layer-by-layer pretraining, regardless of the specific task. Therefore, the high-order features extracted from the hidden layer can be shared with other tasks. The model stacking process is as follows.

1. The input layer of the model is used as the input layer of the first automatic encoder to train the first noise reduction automatic encoder
2. Add a new hidden layer and output layer to train the next automatic encoder
3. Repeat step (2) to get the model with desired depth

The training of automatic encoder model adopts back propagation algorithm. As the loss function of the automatic encoder is the reconstruction error between the output and the input, the output is as close as possible to the input value. For a training sample (*x*, *y*), the loss function is

(1) $$\begin{array}{c} J\left(W,b;x,y\right)=\frac{1}{2}{\left\|h_{W,b}\left(x\right)-y\right\|}^{2}. \end{array}$$

This moment *y*=*x*.

RETRACTED

Random initialization can invalidate symmetry, and then the parameter *W*, *b* is optimized by using optimization algorithm such as batch gradient descent. In gradient descent method, each iteration updates the parameters as follows:

(2) $$\begin{array}{c} W_{ij}^{\left(l\right)}=W_{ij}^{\left(l\right)}-\alpha \frac{\partial }{\partial W_{ij}^{\left(l\right)}}J\left(W,b\right),\\ b_{i}^{\left(l\right)}=b_{i}^{\left(l\right)}-\alpha \frac{\partial }{\partial b_{i}^{\left(l\right)}}J\left(W,b\right). \end{array}$$

*α* is the learning rate.

EA is a skill with creative characteristics and creativity of self-development and self-realization. EA is a kind of behavior transaction method closely combined with personality tendency and characteristics. It is the generalisation of EA knowledge and skills, and the major routes are “innovation consciousness” and “EA,” which strengthen cooperation in Industry-University-Research, invite and introduce industry enterprises to participate in practice teaching and general practice teaching, systematically optimize the design, ensure the controllability and effectiveness of practice teaching, and establish a practical, scientific, and multilevel practice teaching system. To sum up, the path of entrepreneurship education factors to EA formation is shown in Figure 1.

The development of an innovative personality and the system for supporting IEE are examples of recessive environmental factors. This variable primarily captures the impact of the subtle and covert environment on the development of EA talent. Its duties include protecting and promoting IEE through system building and cultural environment construction, guiding and encouraging innovation consciousness and entrepreneurship, and so on. In order to cultivate fundamental intelligence and creative EA ability, the teaching process of professional education must be capable of all-intelligence training. This requires adjusting the teaching methods and evaluation methods. To develop college students' innovative EA is at the heart of establishing the talent training mode and goal in universities, implementing IEE, and cultivating IEE consciousness and spirit [16].

RETRACTED

The model learning process consists of two stages: calculation feedforward and back propagation, and the tanh function is used as the activation function of the two hidden layers. This allows the model to automatically learn the semantic features of the context. Due to the following characteristics of the tanh derivative,

(3) $$\begin{array}{c} \frac{\text{d}}{\text{d}x}\tanh\left(x\right)=1-\;\tanh^{2}\left(x\right). \end{array}$$

This feature makes it easier for the network to calculate the gradient when propagating back.

The process of model training is to use the labeled training sample (*x*^(*i*)^, *f*^(*i*)^) to train the model and find the parameter set *θ*, so as to maximize the log-likelihood probability with regular terms. The likelihood function is as follows:

(4) $$\begin{array}{c} L\left(\theta \right)=\sum_{i=1}^{N}\log\;p\left(f^{\left(i\right)}|x^{\left(i\right)},\theta \right)+R\left(\theta \right). \end{array}$$

Here, *N* is the number of training samples, *x*^(*i*)^ is the *i* th training sample, *f*^(*i*)^ is the frame of the target word in the *i* th sentence, and *R*(*θ*) is the regularization term to prevent overfitting. In the training process, the random gradient ascending method is used to learn the parameters in the likelihood function.

### 3.2. Design of EA Evaluation Model for College Students

In the new era, it is especially important for college students to have team spirit and team cooperation consciousness for entrepreneurial success. From this perspective, college students' mental health education can help college students to know their mental health level, know themselves better, make an accurate self-orientation, help college students to be clear and practical, and help them develop their potential. Group psychological counselling in college students' mental health education is not out of date for contemporary college students. It combines ability with team goals and improves the quality of team cooperation required by society.

In the process of educating people about mental health, we should combine the needs of innovative EA and innovative and enterprising personality and pay attention to developing students' innovative thinking, creating harmonious interpersonal relationships, managing emotional pressure and emotional intelligence, and establishing a good self-awareness to form a good self-awareness and a positive attitude. A number of training units in personal development, innovative thinking, interpersonal communication, teamwork, and emotional stress management can be created by psychological counselling for innovative and entrepreneurial groups when combined with the training content of psychological quality for innovative and entrepreneurial groups. Additionally, by taking the temperament type test, students can gain a better understanding of their temperament types, play to their strengths, and avoid their weaknesses in IEE activities.

RETRACTED

BPNN (BP neural network) refers to the multilayer perceptron network model trained by BP algorithm, which is a widely used feedforward neural network model. According to the actual needs, each neuron can choose the appropriate transfer function and output function. Neural network is highly adaptive, self-organizing, and self-learning. According to the laws and characteristics of functions, neural networks can scientifically and reasonably analyze complex problems and find the most effective strategies and methods to solve them, as shown in Figure 2.

The difference between neural network models lies in the difference of transfer functions, which leads to the difference of information processing methods. The application of BPNN optimization is to continuously optimize the weights or thresholds until the output error of the network reaches the minimum value. The objective function is as follows:

(5) $$\begin{array}{c} E\left(k\right)=\frac{1}{2}\sum_{i=1}^{n}\sum_{j=1}^{m}{\left[t_{ij}-a_{ij}\left(k\right)\right]}^{2}, \end{array}$$

*n* is the number of input vectors and *m* is the number of output vectors.

The weight correction process is as follows:

(6) $$\begin{array}{c} x\left(k+1\right)=x\left(k\right)-\text{ag}\left(k\right),\\ g\left(k\right)=\frac{\partial E\left(k\right)}{\partial x\left(k\right)}, \end{array}$$

*t* is the iteration quantity; *x*(*k*) is the interlayer connection weight or threshold vector after *k* iterations; *g*(*k*) is the gradient vector of network error after *k* iterations; *α* is the learning rate; *E*(*k*) is the total mean square error between the expected output and the actual output after *k* iterations.

BPNN is a multilayer feedforward network, which solves the basic principle of integral evaluation: the characteristic information of the evaluation object must be collected in advance and converted into the input vector of the neural network, and the corresponding integral evaluation is only used as the output of the neural network. Neural network can be regarded as a tool with qualitative and quantitative functions, and the objects of comprehensive evaluation can cover objects other than samples.

The input layer belongs to the front part, the hidden layer belongs to the middle part, and the output layer belongs to the end part, which together form BPNN.

(7) $$\begin{array}{c} o_{k}=f\left({\text{net}}_{k}\right),\;k=1,2,\ldots ,n,\\ {\text{net}}_{k}=\sum_{j=o}^{m}w_{jk}y_{j},\;k=1,2,\ldots ,n. \end{array}$$

RETRACTED

#### 3.2.1. Transfer function

(8) $$\begin{array}{c} \log\text{ sig}\left(x\right)=\frac{1}{1+e^{-x}},\\ \tan\text{ sig}\left(x\right)=\frac{2}{1+e^{-2x}}-1. \end{array}$$

Layer by layer, starting at the input layer and moving through the hidden node layer before reaching the output layer, is how the forward propagation process works. The error signal is reduced by adjusting how much each layer's neurons are connected to one another. The process flow diagram for the student EA evaluation is shown in Figure 3.

The input data, such as network convergence time value, network initialization value, students' academic performance, ideological and moral ability value, physical and mental health ability value, and personal ability value, are evaluated by network algorithm in turn. Once the decision is successful, the expert system will display the evaluation results to the users and write the relevant information of these evaluations into the mining database, including the names and numbers of students selected as the evaluation objects. If the classification analysis produces some new rules, learn the conditions of these rules in the mining database, so as to prepare for adding new decision information in the expert knowledge base in the future.

In the fields of innovation and business education, the unique personality has received sufficient attention; therefore, from the perspective of student development, based on the theory of personality education, we should cultivate students' complete personalities, explore their potential and intelligence, and then give your due intuition full play. Through testing, psychology instructors can assist students in understanding their aptitudes and personality traits in developmental counselling. They can also provide them with individualised advice and support to help them develop their aptitudes and personalities to their full potential. In our deliberations, we should focus on fostering students' innovative psychological qualities and laying the groundwork for their development.

## 4. Experiment and Results

In order to test the feasibility of the evaluation model, some students of *C* University were selected as the survey objects, and the EA status of college students was analyzed. Validity is used to analyze whether the research project is reasonable and significant. Validity analysis adopts the data analysis method of factor analysis, and comprehensive analysis is carried out by variance explanatory rate value, factor load coefficient value, and other indicators to test the validity of the data. In this study, principal component analysis is used to extract the common factor, and the maximum variance method is used to rotate the factor, and the results are shown in Figure 4. The rotated factor load matrix data is obtained through analysis, as shown in Figure 5.

RETRACTED

The results show that three factors can be extracted to evaluate college students' EA. Among them, factor 1 consists of 4–7 items, reflecting the basic qualities of college students' EA, and the other 2 factors consist of 8–10 items, reflecting the general EA ability of college students. According to the previous reliability and validity analysis results, it can be seen that the scale of EA evaluation questionnaire for college students has passed the reliability and validity test, so the reliability and validity of the questionnaire are good.

It can be concluded that among the three evaluation dimensions of college students' EA, the basic quality, which is the core skill, has the highest score, followed by general skills and professional skills, with a small gap between them. Although the comprehensive evaluation result is “good,” there is still a certain gap with the excellent level. This study holds that motivation consciousness is a psychological state. Instant business motivation or business awareness cannot have an effective impact on all business activities. Therefore, in order to form a long-term spontaneous entrepreneurial desire and incentive tendency, university, as the main implementers of EA training for college students, must reform the mode of entrepreneurship education.

The whole EA questionnaire for college students is divided into three parts: professional ability, method ability, and social ability. In this section, in addition to general descriptive statistics, “max” and “min” are introduced, which represent the maximum and minimum scores that can be obtained in this section. The average EA of college students in *C* University is 7.18, as shown in Table 1.

In general, students at *C* University are more methodologically adept than they are in terms of their professional and social abilities. It is evident that students at *C* University are more skilled at problem-solving and analysis. The lowest professional ability and smallest standard deviation are, in relative terms, found among students at *C* University. The difference between students is not very wide, as can be seen. College students can practise their social skills in a variety of ways, including by joining clubs, getting along with their roommates and classmates, and forming teams to complete tasks or compete in events. Students at *C* University have better social skills than professional ones, for this reason. However, it is not as strong as method ability, which explains why most of the students in school major in science and engineering and why problem-solving is done in a more logical manner. Because of this, the student's interpersonal abilities fall short of his mastery of methodology.

RETRACTED

The author believes that there is a significant negative correlation between spirituality and social entrepreneurship; that is, the less obvious the personality traits of spirituality, the stronger the social entrepreneurship of students. Introversion is positively correlated with social EA; that is, the more extroverted students are, the higher their social EA is. In order to further investigate the partial correlation coefficient analysis of personality traits and specific indicators of social ability, Table 2 is the partial correlation coefficient table of the components of entrepreneurial social ability and personality traits of *C* University students.

Generally speaking, apart from “the ability to adapt to change and bear setbacks,” spiritual quality is negatively correlated with the other four dimensions of social ability, among which it is significantly negatively correlated with “interpersonal skills” and “cooperation skills.” The author believes that students with low psychological quality have good interpersonal skills, high emotional intelligence, and strong adaptability to the environment, so their interpersonal skills and cooperation skills are stronger in the dimension of social skills. People with low psychological quality are good at communication, and they are also willing to find their own shortcomings through communication. They can accept others' opinions and suggestions modestly, not be self-centered and correct them in time. This will enable students to better integrate into the team, cooperate with others, and achieve a win-win situation.

Taking the trained BPNN as a practical evaluation tool, the BPNN model becomes the evaluation model of students' IEE, determining the number of neurons in hidden layer and output layer. The actual output value of the network is unique, so the number of neurons in the output layer is also unique. By comparing the number of neurons in the hidden layer with those in the input layer and the output layer, it is vulnerable to interference and conflict from the surrounding environment. The relationship between the number of hidden layer neurons and the error is shown in Figure 6. The relationship between the number of hidden layer neurons and the maximum error value is shown in Figure 7.

When analyzing the number of neurons in the hidden layer, the values are 3, 4, 5, 6, 7, 8, 9, 10, 11, 12, and 13. At this time, the training error is decreasing, but there is a connection. When the test error is 10, 11, and 12, it will first rise and then fall. Generally, the number of neurons in the hidden layer is 11, which is the best choice.

RETRACTED

In order to compare the gradient descent method and the quasi-Newton method in terms of iteration count, network error, generalisation, and prediction accuracy, this paper uses the LM (Levenberg-Marquardt) algorithm. It is important to choose parameters consistently. The total mean square error network serves as the target function for the 8-14-1, which conceals a single-layer BP network with a maximum iteration limit of 1000 and a default target error of 0. The weighted average of the weights acquired using the combination of AHP and coefficient of variation is the anticipated outcome. Each index's weight is calculated by adding professional judgement to the initial data of the evaluation object as well as objective reality. The outcome is more accurate when compared to summation and averaging.

The enhanced BPNN training is finished, and in accordance with the analysis in Figure 8, some test data are randomly chosen to test the BPNN model. Students are then asked to provide the corresponding evaluation values of IEE. The maximum relative error is 1.6 percent, which is roughly close to the ideal state, and the actual value is valid, the expected value is reasonable, and the maximum relative error is valid. The actual value after neural network training is basically consistent with the expected value.

National laws and the scientific and orderly development of entrepreneurship are inextricably linked. A logical and compatible legal framework for college students' IEE should be developed by the national legal department, and local governments should also develop a number of safety precautions that take into account local circumstances and address creation, financing, and training and establish a solid external business environment, start from scratch, and support college students' development as entrepreneurs. This can develop the critical and creative thinking skills of college students and inspire them to pursue IEE. We can provide more plentiful and varied educational resources for college students' independent learning by using data analysis technology to understand their learning needs and laws. IEE is a broad field that encompasses sociology, pedagogy, psychology, and other related disciplines [4], so it is important to create a top-notch teaching staff that is “double-qualified.” The addition of appropriate group psychological counselling to IEE can help students' entrepreneurial psychological qualities, ensure that they have a clear sense of who they are before starting a business, learn to control and manage their emotions when starting a business, know how to handle the pressure of setbacks and failures, and have realistic expectations and well-defined future plans.

RETRACTED

## 5. Conclusions

EA has a larger scope and audience when applied to college students. It is crucial for every college student because it is a higher-level professional skill. This paper examines the relationship between IEE courses and the mental health education of college students from the viewpoints of classroom instruction, daily activities, and mechanism construction. This study defines the content and scope of the study, explains the pertinent theories of EA and skill evaluation, and then conducts a fair assessment of students' IEE using the BPNN model. The BPNN algorithm that is presented in this paper possesses the traits of quick convergence and potent learning capacity. The model's actual value in the simulation experiment is efficient, and the expected value is reasonable. The greatest difference in relative error between them is 1.6 percent, which is essentially the state of nature. It can offer suggestions for improvement, reflect the evaluation of teaching quality objectively, and foster exceptional talent.

## Figures and Tables

**Figure 1:** EA influencing factors influencing path.

**Figure 2:** Topological structure diagram of BPNN model.

**Figure 3:** EA student evaluation program flowchart.

**Figure 4:** Population explanatory variance.

**Figure 5:** The rotated factor load matrix.

**Figure 6:** Relationship between the number of hidden neurons and error.

**Figure 7:** Relationship between the number of hidden neurons and the maximum error.

**Figure 8:** Comparison between expected value and actual value.

**Table 1:** Descriptive statistics of college students' EA status in *C* University.

	Max	Min	Minimal	Maximum	Mean value	Standard deviation
Ability dimension	15	3	3	12	4.33	1.36
Professional competence	15	3	3	10	7.24	3.25
Method ability	15	3	3	8	7.03	2.07
Social competence	15	3	3	8	7.55	2.66
EA	15	3	3	9	7.18	2.53

**Table 2:** Partial correlation coefficient between components of entrepreneurial social ability and personality traits of college students.

Inscape	Spirit quality	Nervous temperament	Internal and external tendencies	Concealment
Ability to withstand setbacks	0.235	−0.886	−0.328	0.221
Interpersonal skills	−0.726	−0.632	0.622	0.206
Negotiation ability	−0.386	−0.332	0.769	0.168
Cooperative ability	−0.801	−0.761	−0.395	0.184
Self-restraint ability	−0.536	0.303	−0.665	0.196

## Data Availability

The data used to support the findings of this study are available from the corresponding author upon request.
